# Fuzi-Lizhong Decoction Alleviates Nonalcoholic Fatty Liver Disease by Blocking TLR4/MyD88/TRAF6 Signaling

**DOI:** 10.1155/2022/1637701

**Published:** 2022-08-26

**Authors:** Jiayao Yang, Ying Zhang, Hongfeng Yi, Yan Liao, Lei Shu, Shu Zhang, Chenyu Li, Liu An, Nianlong Du, Zhaohong Shi, Wei Ma

**Affiliations:** ^1^Department of Gastroenterology, Wuhan Integrated TCM and Western Medicine Hospital, Wuhan, China; ^2^Department of Traditional Chinese Medicine, Hubei University of Traditional Chinese Medicine, Wuhan, China

## Abstract

**Background:**

Fuzi-Lizhong decoction (FLD) derives from the ancient Chinese Pharmacopoeia and has been clinically used for years. The present study aimed to investigate the activities and underlying mechanisms of FLD against nonalcoholic fatty liver disease (NAFLD).

**Methods:**

*In vivo* studies were conducted by inducing NAFLD in rats with a high-fat diet, and *in vitro* studies were performed on HL-7702 cells treated with oleic and linoleic acids. Total cholesterol (TC), triglyceride (TG), and blood glucose (Glu) levels were detected using an automatic biochemical analyzer. The expression of IL-2, IL-6, and TNF-*α* in sera and cell culture supernatants was measured by ELISA. The mRNA and protein levels of TLR4, MyD88, and TRAF6 were measured in liver tissue and HL-7702 cells using reverse transcription-quantitative polymerase chain reaction and western blot.

**Results:**

FLD significantly reduced the TC, TG, Glu, FFA, IL-2, IL-6, and TNF-*α* levels in NAFLD rats and HL-7702 cells. Analysis of liver lipid content by Oil Red O staining revealed a significant increase in hepatic lipid accumulation in rats with NAFLD, but this lipid accumulation was reversed by FLD treatment. In addition, the mRNA expression levels of TLR4, MyD88, TRAF6, and NF-*κ*B p65 as well as the protein levels of TLR4, MyD88, TRAF6, and NF-*κ*B p65 were decreased after FLD treatment. FLD significantly reduced inflammation and improved collagen accumulation *in vivo* and *in vitro* by inhibiting the activation of the TLR4/MyD88/TRAF6 signaling pathway.

**Conclusions:**

FLD exerted potent protective effects against NAFLD via TLR4/MyD88/TRAF6 signaling. These findings provide novel insights into the mechanisms whereby this compound acts as an anti-inflammatory agent and highlight the potential application of FLD in the treatment of acute liver failure (ALF).

## 1. Background

The recent increase in fat intake due to improvements of living standards has resulted in an increase in the incidence of nonalcoholic fatty liver disease (NAFLD), particularly in younger patients in countries such as China [1–3]. NAFLD is a medical condition characterized by a series of hepatic pathological changes, including simple steatosis, nonalcoholic steatohepatitis, and cirrhosis [4,5]. The pathogenesis of NAFLD is an orchestrated multistep process in response to hepatic lipid accumulation and oxidative stress. It has been demonstrated that approximately 15% of NAFLD cases may result in cirrhosis and even hepatocellular cancer [6,7]. In affluent regions of China, the incidence of NAFLD is approximately 15% [8]. An appropriate nutritional intake and exercise are recommended to prevent excessive body weight; however, this health problem caused by overnutrition has not yet been conquered. Therefore, new strategies are required to reduce the risk of NAFLD.

The innate immune system is closely related with NAFLD progression. Several studies have described a close association between NAFLD development and many pathogenic events such as activation of the innate immune system and hepatic macrophage recruitment, which cause changes in lipid homeostasis [9,10]. Toll-like receptors (TLRs) are pattern recognition receptors that recognize pathogen-associated molecular patterns and allow the host to detect microbial infection [11]. TLRs may be involved in NAFLD by regulating innate and adaptive immune responses [12]. TLR4 is the receptor for lipopolysaccharide (LPS); it can trigger two different signaling pathways, a myeloid differentiation factor 88 (MyD88)-dependent pathway that results in the activation of nuclear factor *κ*B (NF-*κ*B) and TNF receptor-associated factor 6 (TRAF6), and an MyD88-independent pathway requiring the Toll/interleukin-1 receptor (TIR)-containing adaptor molecule [13]. The activation of TLR4 pathways can stimulate downstream signaling cascades, resulting in the production of proinflammatory cytokines, chemokines, and type I interferon. Moreover, the activation of TLR4 signaling might be disturbed at multiple steps during the initiation and progression of NAFLD [14].

Fuzi-Lizhong decoction (FLD) is a Chinese herbal concoction consisting of *Panax ginseng* C.A. Mey., *Aconitum carmichaeli Debx*., *Glycyrrhiza inflata* Bat., *Atractylodes macrocephala* Koidz., and *Zingiber officinale* Rosc. FLD has significant therapeutic effects on dyspnea caused by chronic obstructive lung disease as well as pulmonary oedema provoked by heart failure and inflammation of the viscera, clearly relieving various symptoms of respiratory and myocardial diseases [15–17]. However, the effect of FLD on liver disease has rarely been reported. In the present study, we used a high-fat and high-fructose diet to establish a suitable animal model of NAFLD and explored the effect and potential mechanisms of FLD on NAFLD.

## 2. Methods

### 2.1. Reagents and Materials

FLD is composed of Radix Codonopsis (15 g), Rhizoma Atractylodis Macrocephalae (9 g), Radix Glycyrrhizae (6 g), Rhizoma Zingiberis (9 g), and Radix Aconiti Lateralis Preparata (9 g). Herbs were purchased from Hubei Tianji Chinese Herbal Sliced Medicine Co., Ltd. The decoction was carried out according to the method described by Yang Xin [18]. Polyene phosphatidylcholine was purchased from Sanofi Beijing pharmaceuticals Co., Ltd (Cat No. 5JD065 B). IL-2 (RA20132), IL-6 (RA20607), and TNF-*α* (RA20035) ELISA kits were purchased from Bioswamp (Wuhan, China). The antibiotic (penicillin and streptomycin) and antimycotic (amphotericin B) solutions were obtained from Sigma-Aldrich (USA). TLR4 (ab13867, 1 : 1000 dilution), NF-*κ*B p65 (ab16502, 1 : 2000 dilution), p-NF*κ*B (ab86299, 1 : 2000 dilution), MyD88 (ab2064, 1 : 1000 dilution), and TRAF6 (ab33915, 1 : 5000 dilution) antibodies were purchased from Abcam (USA). Anti-GAPDH antibody (2118, 1 : 10000 dilution) was purchased from CST (USA). The feed for a normal diet (MD17121) was obtained from Jiangsu Medison Biomedical Co. Its main nutrients are shown in Table 1.

### 2.2. Animals and Experimental Groups

Forty-eight male Wistar rats were obtained from Hubei Provincial Academy of Preventive Medicine (certification No. 42000600013948). Rats were housed in a specific pathogen-free facility at Wuhan First Hospital. Following an acclimatization period, rats were divided into two groups: a control group (CON, *n* = 8) receiving a standard diet and saline by oral gavage for four weeks, and a model group (*n* = 40) receiving a high-fat diet (standard laboratory diet + 2% cholesterol + 10% lard + 2.5% vegetable oil) [19,20] for four weeks. The model group was then randomly divided into five groups (*n* = 8 each): a NAFLD model group (MOD), a positive control group (PC, treatment with 30 mg/kg/d polyene phosphatidylcholine), and FLD groups (treatment with 5, 10, and 20 g/kg/d FLD). Rats were maintained under a 12 h light-dark cycle at 23 ± 2°C. After the experiment, the rats were euthanized by intraperitoneal injection of 200 mg/kg pentobarbital, packaged, and eventually burned. All experimental procedures were approved by the Animal Ethics Committee of Wuhan Integrated TCM and Western Medicine Hospital (certificate no. 42000600013948).

### 2.3. Blood Collection and Processing

At the end of the experiment, pentobarbital was injected intraperitoneally at 40 mg/kg, blood was collected from the abdominal aorta after anesthesia and anticoagulated with heparin, and the serum was isolated and reserved.

### 2.4. Cell Culture and Treatment

The human liver HL-7702 cell line was obtained from Procell (CL-0111). HL-7702 cells were cultured in Dulbecco's modified Eagle's medium (DMEM) supplemented with 10% FBS (ThermoFisher, Waltham, USA), 100 U/mL penicillin, 100 mg/ml streptomycin, and 100 mg/ml amphotericin B. The cells were grown in an incubator with a humidified atmosphere (95% air/5% CO_2_ v/v) at 37°C for 48 h until 80% confluence and then washed. The test was divided into six groups: a control group incubated with an equal amount of medium as a control for 48 h; a model group incubated with 1 ml/l of fat emulsion (20%) for 48 h; FLD intervention groups (low, medium, and high) incubated with 1 ml/l of fat emulsion (20%) + low (0.5 g/ml), medium (1.0 g/ml), and high (1.5 g/ml) doses of FLD for 48 h; and a positive control group cultured with 1 ml/l of fat emulsion (20%) + polyene phosphatidylcholine (5 *μ*mol/l) for 48 h.

### 2.5. Histological and Serological Examinations

Liver tissues were fixed in 4% paraformaldehyde for 30 min and stained by 0.5% Oil Red O. The stained sections were observed under a microscope (Olympus CX31-LV320, Tokyo, Japan). The serum total cholesterol (TC), triglyceride (TG), and blood glucose (Glu) levels were detected using an automatic biochemical analyzer (model 7180, Tokyo, Japan). Free fatty acid (FFA) levels were detected by a non-esterifiedfFree fatty acids assay kit (A042-1, Nanjing Jiancheng, Nanjing, China).

### 2.6. ELISA

IL-2, IL-6, and TNF-*α* levels in the serum or cell culture supernatants were evaluated by ELISA kits and the assays were performed in accordance with the manufacturer's protocols.

### 2.7. Total RNA Extraction and Reverse Transcription-Quantitative Polymerase Chain Reaction (RT-qPCR)

Total RNA was extracted from liver tissue or HL-7702 cells using TRIzol reagent (Takara Bio Inc., Dalian, China) and assessed using an ultraviolet spectrophotometer (Nanodrop 2000, Thermo) and 1% agarose electrophoresis (DYC-31D, BIO-RAD). For each sample, 1 *μ*g RNA was reverse transcribed to obtain first-strand cDNA using the PrimeScript® RT reagent kit with gDNA Eraser (Takara Bio, Inc.) as per the manufacturer's instructions. The reaction mixture (20 *μ*l total volume) contained 10 *μ*l 2 X SYBR Premix Ex Taq™ (Takara Bio, Inc.), 0.5 *μ*l of each primer, and 0.2 ± 0.02 *μ*g cDNA template. The following three-step qPCR reaction was performed: predenaturation at 95^o^C for 30 sec, followed by 40 cycles, including denaturation at 95°C for 3 min and annealing at 60^o^C for 20 sec, and elongation at 72°C for 20 sec. The primers used are shown in Table 2. Gene expression levels were then calculated using the 2^−ΔΔCq^ method. For each group, three samples were measured and three technical replicates of each measurement were obtained.

### 2.8. Western Blot

Protein expression levels were analyzed by western blot and conducted using standard methods with modifications. Liver tissue samples were homogenized in RIPA lysis buffer containing protease inhibitor at 4°C. For *in vitro* experiments, cells were washed twice with phosphate-buffered saline (PBS) and lysed with RIPA buffer (Beyotime, China) containing protease inhibitor at 4°C. Both cell and tissue lysates were centrifuged at 12000 × *g* for 15 min, and the supernatants were collected. Protein concentration was detected using a BCA kit (Bio-Swamp Life Science). Equal amounts of protein (30 *μ*g) were separated by 10% SDS-polyacrylamide gel and then transferred onto a PVDF membrane (EMD Millipore, Billerica, MA, USA). Membranes were blocked for 2 h at room temperature with 5% skim milk in Tris-buffered saline (20 mmol/l Tris, 500 mmol/l NaCl, and 0.05% Tween 20). Subsequently, the membrane was incubated with primary antibodies. GAPDH was used as an internal reference. Membranes were subsequently washed with Tris-buffered saline and incubated with goat antirabbit secondary antibody conjugated to horseradish peroxidase (Cat No. W4011; dilution, 1 : 3000; Promega Corporation, Madison, WI, USA) for 2 h at room temperature. Immunoreactivity was visualized via a colorimetric reaction using enhanced chemiluminescent substrate buffer (EMD Millipore). Membranes were analyzed using a Gel Doc EZ imager and bands were quantified using Quantity One 5.0 (Bio-Rad Laboratories, Hercules, CA, USA).

### 2.9. Experimental Outcomes

We used the effect of FLD on TLR4/MyD88/TRAF6 signaling in rat livers and HL-7702 cells as the primary experimental outcomes. The levels of inflammatory factors and hepatic lipid contents were used as secondary experimental outcomes.

### 2.10. Statistical Analysis

Differences between the means of the experimental groups were evaluated by analysis of variance (ANOVA) using the SPSS 19.0 software package. Statistical significance was set at *P* < 0.05. All results were expressed as mean ± SD.

## 3. Results

### 3.1. Effects of FLD on Serum Levels and Hepatic Lipid Contents in Rats with NAFLD

All animals in this study were healthy before and after treatment, and without death and adverse events. To evaluate the treatment effect of FLD on NAFLD, lipid accumulation, serum levels of TC, TG, and Glu, and FFA levels in liver tissue were compared between the groups. TC, TG, Glu, and FFA levels were significantly increased in the MOD group compared to those in the CON group. Compared to the MOD group, the FLD groups had significantly decreased TC, TG, Glu, and FFA levels (Figure 1(a)). Analysis of the hepatic lipid contents by Oil Red O staining revealed that hepatic lipid accumulation (red fat drops) increased significantly in the MOD group, and that lipid accumulation was reversed by FLD treatment (Figure 1(b)).

### 3.2. FLD Treatment Reduces the Levels of Inflammatory Factors in the Serum and the Liver of Rats

As shown in Figure 2, the serum and liver levels of IL-2, IL-6, and TNF-*α* were markedly increased in the MOD group compared with those in the CON group. Moreover, these increases were significantly attenuated by FLD administration.

### 3.3. FLD Treatment Attenuates the Activation of TLR4/MyD88/TRAF6 Signaling in Rat Livers

As shown in Figure 3(a), the mRNA expression levels of TLR4, MyD88, TRAF6, and NF-*κ*B p65 in the MOD group were conspicuously increased compared with those in the CON group, and were all significantly decreased by FLD treatment. The livers from the rats in the MOD group exhibited drastically increased hepatic protein levels of TLR4, MyD88, and TRAF6, whereas FLD treatment significantly decreased the levels of all these molecules (Figure 3(b)). In addition, the activation of NF-*κ*B p65 in the livers of the MOD group was significantly inhibited by FLD treatment (Figure 3(c)). Together, these data indicated that FLD attenuates NAFLD by blocking TLR4/MyD88/TRAF6 signaling.

### 3.4. FLD Reduces the Levels of IL-2, IL-6, and TNF-*α* in HL-7702 Cells

To verify the treatment effect of FLD, a NAFLD cell model was induced in HL-7702 cells [21,22], and the cells were exposed to different doses of FLD. The IL-2, IL-6, and TNF-*α* levels in cell supernatants are shown in Figure 4. Compared with those in the CON group, the levels of IL-2, IL-6, and TNF-*α* increased significantly in the MOD group, whereas FLD treatment decreased the levels of all these molecules.

### 3.5. FLD Inhibits the Activation of TLR4/MyD88/TRAF6 Signaling in HL-7702 Cells

The protein and mRNA expression levels of TLR4, MyD88, and TRAF6 as well as the mRNA expression levels of NF-*κ*B p65 in HL-7702 cells were used to evaluate the effect of FLD on NAFLD cells, and the results are shown in Figure 5. The protein and mRNA expression levels of TLR4, MyD88, and TRAF6 as well as the mRNA expression levels of NF-*κ*B p65 in model cells were markedly increased compared with those in normal control cells, whereas FLD treatment decreased the expression levels of all these molecules.

## 4. Discussion

NAFLD is a passive and irreversible pathological process induced by the necrosis of liver parenchymal cells, and recent evidence has shown that even advanced fibrosis is reversible [23]. Therefore, the development of novel and effective treatment strategies to reverse NAFLD is of critical importance. In the present study, FLD showed significant effects against NAFLD as evidenced by the decreased TC, TG, Glu, and FFA levels and the alleviation of histopathological changes. Furthermore, FLD was effective in suppressing TLR4/MyD88/TRAF6 signaling to inhibit the release of the inflammatory factors IL-2, IL-6, and TNF-*α in vivo* and *in vitro*.

Hepatic inflammation is tightly related to liver disease. Chronic activation of the inflammatory pathways has been shown to promote hepatocarcinogenesis [24]. During the progression of NAFLD, TLR4 signaling is involved in liver injury and repair-related functions [25]. The present study illustrated that TLR4/MyD88/TRAF6 signaling is significantly activated in NAFLD rats. TLR4 signaling is activated in rats in which nonalcoholic hepatitis (NASH) is induced by a choline-deficient L-amino acid-defined diet, resulting in the up-regulation of TNF-*α* expression, which suggests that TLR4 might induce further liver injury [26]. In this study, the activation of TLR4/MyD88/TRAF6 signaling in NAFLD rats was blocked by FLD administration. Proinflammatory cytokines including IL-1, IL-6, and TNF-*α* are released from inflammatory cells, and their levels are strictly regulated by proinflammatory and anti-inflammatory responses [27]. In these processes, NF-*κ*B plays a critical role in the regulation of inflammatory responses by affecting the production of various proinflammatory cytokines such as IL-1, IL-2, IL-6, and TNF-*α* [28,29]. In this study, the anti-inflammatory capability of FLD mainly resulted from the decreased IL-2, IL-6, TNF-*α*, and NF-*κ*B p65 levels via the reduction of TLR4/MyD88/TRAF6 signaling *in vivo* and *in vitro*.

FLD has been used in the clinical treatment of some diseases, such as pulmonary and heart disease, for hundreds of years. Twenty-one constituents have been identified in Fuzi-Lizhong by ultraperformance liquid chromatography with time-of-flight mass spectrometry, including ginsenoside Rb1, mesaconitine, aconitine, salsolinol, and glycyrrhizic acid [30]. Ginsenoside was determined to be the most compound of P. ginseng, and showing anti-inflammatory effects by inhibiting the activation of NF-κB. [30]. In addition, aconitine exerts anti-inflammatory effects by suppressing TNF-*α* and NF-*κ*B activation [31,32]. Furthermore, ginsenoside can improve inflammatory disease by inhibiting IRAK-1 activation via TLR-4 and MAPK signaling [33]. In the present study, the expression of TNF-*α* and NF-*κ*B was significant decreased by FLD in NAFLD rats, indicating that FLD can attenuate NAFLD by inhibiting the inflammatory response.

In conclusion, our findings suggest that FLD may attenuate NAFLD through its effects on TLR4/MyD88/TRAF6 signaling. FLD inhibited the activation of TLR4/MyD88/TRAF6 signaling via down-regulation of TLR4, MyD88, and TRAF6 mRNA and protein levels. The inhibition of NF-*κ*B led to the inhibition of the inflammatory response. Notably, the underlying mechanisms are certainly more complex than what is described here. In addition, our results do not exclude the possible involvement of other signaling pathways and mechanisms in the suppression of NAFLD by FLD. Nevertheless, our findings provide novel insights into the mechanisms whereby FLD acts as a potent anti-inflammatory agent, and suggest that FLD may be used to treat NAFLD. Further experimental data and clinical studies using this traditional Chinese medicine are required to support the present findings.

## 5. Conclusions

FLD exhibited potent protective effects against NAFLD through its action on TLR4/MyD88/TRAF6 signaling. These findings provide novel insights into the mechanisms whereby this compound acts as an anti-inflammatory agent, and highlight its potential use for the treatment of acute liver failure in the future.

## Figures and Tables

**Figure 1:** FLD improves the symptoms of NAFLD. (a) The serum TC, TG, and Glu levels and the liver levels of FFAs were detected by the ELISA kits (*n* = 9). (b) Representative images of Oil Red O-stained liver sections from each group (bars: 100 *μ*m). All values are expressed as the mean ± SD (*n* = 3). ^*∗*^*P* < 0.05 versus NC group; #*P* < 0.05 versus MOD group; ▲*P* < 0.01 versus HIG group.

**Figure 2:** FLD inhibits the production of IL-2, IL-6, and TNF-*α* in the serum and the liver of NAFLD rats. All values are expressed as the mean ± SD (*n* = 9). ^*∗*^*P* < 0.05 versus NC group; #*P* < 0.05 versus MOD group; ▲*P* < 0.01 versus HIG group.

**Figure 3:** FLD inhibits the activation of TLR4/MyD88/TRAF6 signaling in NAFLD rats. (a) The mRNA expression levels of TLR4, MyD88, TRAF6, and NF-*κ*B p65 in rat liver tissue were detected by RT-qPCR. (b) The TLR4, MyD88, and TRAF6 protein levels in rat liver tissue were detected by western blot. (c) The protein levels of NF-*κ*B p65 and p-NF*κ*B in rat liver tissue were detected by western blot. All values are expressed as the mean ± SD (*n* = 3). ^*∗*^*P* < 0.05 versus NC group; #*P* < 0.05 versus MOD group; ▲*P* < 0.01 versus HIG group.

**Figure 4:** The production of IL-2, IL-6, and TNF-*α* by NAFLD HL-7702 cells is inhibited by FLD treatment. All values are expressed as the mean ± SD (*n* = 9). ^*∗*^*P* < 0.05 versus NC group; #*P* < 0.05 versus MOD group; ▲*P* < 0.01 versus HIG group.

**Figure 5:** FLD blocks TLR4/MyD88/TRAF6 signaling in HL-7702 cells. (a) The mRNA expression levels of TLR4, MyD88, TRAF6, and NF-*κ*B p65 in HL-7702 cells were detected by RT-qPCR. (b) The TLR4, MyD88, and TRAF6 protein levels in HL-7702 cells were detected by western blot. All values are expressed as the mean ± SD (*n* = 3). ^*∗*^*P* < 0.05 versus NC group; #*P* < 0.05 versus MOD group; ▲*P* < 0.01 versus HIG group.

**Table 1:** Main nutrient content (content per kg of feed).

Items	Contents
Water content, g≤	100
Crude protein, g≥	180
Crude fat, g≥	40
Crude fiber, g≤	50
Crude ash, g≤	80
Calcium, g	10–18
Total phosphorus, g	6–12
Calcium: total phosphorus	1.2:1–1.7 : 1
Lysine, g≥	8.2
Methionine + cystine, g≥	5.3

**Table 2:** Primer sequences.

Primers	Sequence	Amplified fragment size (bp)
TLR4-F	GAATGAGGACTGGGTG	189
TLR4-R	CAACGGCTCTGGATA	

MYD88-F	TGCCAGAAATACATACGC	108
MYD88-R	GGTGATGCCTCCCAGT	

TRAF6-F	GGAAACGCAGAGCAT	177
TRAF6-R	CCAGGGCTATGAATGA	

NFKB–F	TGCGTTTCCGTTACAAG	154
NFKB-R	TGAGGTGGGTCTTTGGT	

GAPDH-F	CAAGTTCAACGGCACAG	138
GAPDH-R	CCAGTAGACTCCACGACAT	

## Data Availability

The data used to support the findings of this study are included within the article.

## Abbrevations

NAFLD: Nonalcoholic fatty liver disease
TLRs: Toll-like receptors
LPS: Lipopolysaccharide
MyD88: Myeloid differentiation factor 88
NF-*κ*B: Activation of nuclear factor *κ*B
TRAF6: TNF receptor associated factor 6
FLD: Fuzi-Lizhong decoction
DMEM: Dulbecco's modified Eagle's medium
TC: Total cholesterol
TG: Triglyceride
Glu: Blood glucose
RT-qPCR: Reverse transcription-quantitative polymerase chain reaction
ELISA: Enzyme-linked immuno sorbent assay
ALF: Acute liver failure.
